The article "Statin-Induced Autoimmune Necrotizing Myositis: A Case Report" was published in 2022. Journal: Cureus.

# Statin-Induced Autoimmune Necrotizing Myositis: A Case Report

**DOI:** 10.7759/cureus.29475

**Published:** 2022-09-22

**Authors:** Hussein Almadhoun, Nancy Mesiha

**Affiliations:** 1 Department of Internal Medicine, Ascension St. John Hospital, Detroit, USA; 2 Department of Cardiology, Ascension St. John Hospital, Detroit, USA

**Keywords:** statin-induced myosistis, guideline-directed medical therapy, cardiovascular disease, high-statin therapy, statin-induced myopathy, statin-induced necrotizing autoimmune myopathy

## Abstract

Statin therapy is considered one of the main therapies indicated to reduce the risk of cardiovascular death in patients with atherosclerotic cardiovascular disease. Maximal risk reduction is linked to the degree of reduction of the low-density lipoprotein cholesterol; therefore, high-intensity dosing is required with coronary artery disease. Musculoskeletal side effects are reported with the use of statin, especially at high doses. Although myopathy is a common side effect, autoimmune-mediated necrotizing myositis is a rare side effect usually related to the development of hydroxymethylglutaryl-coenzyme A reductase antibodies which attack the muscles leading to swelling manifesting as muscle weakness and pain, as presented in our case report.

## Introduction

Statin therapy is considered one of the cornerstones in the treatment of patients with coronary artery disease for its benefit in reducing the incidence of cardiovascular death, myocardial infarction (MI), stroke, and recurrent ischemic events. The magnitude of the benefit is related to the low-density lipoprotein cholesterol (LDL-C) lowering effect, and, therefore, high-intensity dosing is recommended [1]. Musculoskeletal side effects are well-established [2]. Myopathy and myositis have been reported as side effects due to statin therapy, with myositis being less reported. Here, we present the case of a patient with statin-induced necrotizing myositis after about four months of statin use.

## Case presentation

A 57-year-old female presented with a chief complaint of bilateral arm and leg weakness for three days, which was constant and progressively worsening. The patient reported that she was not able to lift herself from the toilet and most of the weakness was in her thighs. She reported two falls recently related to not being able to get up. The patient had a medical history significant for coronary artery disease with a percutaneous coronary intervention in the past. She was chronically on rosuvastatin 40 mg daily for this indication and reported a history of myopathy in the past. In addition, she reported a history of angiotensin-converting enzyme (ACE)-inhibitor-induced angioedema leading to prior intubation and tracheostomy. She denied excessive alcohol use. Initial labs showed a significant creatine phosphokinase (CPK) level elevated at 10,919 IU/L, and an erythrocyte sedimentation rate (ESR) >120 mm/hour. Creatinine was elevated at 3.55 mg/dL with a prior baseline of 1.1 mg/dL, and the thyroid-stimulating hormone (TSH) level was normal. Given the proximal thigh weakness and the elevated CPK, a decision was made to obtain magnetic resonance imaging (MRI) of bilateral thighs (Figure 1). MRI showed symmetrical edema involving the proximal and mid-thigh muscles. The initial extended myositis panel was negative, as shown in Table 1.

The article "Statin-Induced Autoimmune Necrotizing Myositis: A Case Report" was published in 2022. Journal: Cureus.

**Figure 1:** Magnetic resonance imaging showing symmetrical edema involving the proximal mid-thigh muscles.

**Table 1:** Extended myositis panel results.

Antibody Tested	Results
SAE1 (SUMO-activating enzyme) antibody	Negative
NXP2 (nuclear matrix protein-2) antibody	Negative
MDA5 (CADM-140) antibody	Negative
TIF-1 gamma (155 kDa) antibody	Negative
Hydroxymethylglutaryl-coenzyme A antibody	Negative
PL-12 (alanyl-tRNA synthetase) antibody	Negative
PL-7 (threonyl-tRNA synthetase) antibody	Negative
OJ (isoleucyl-tRNA synthetase) antibody	Negative
EJ (glycyl-tRNA synthetase) antibody	Negative
Signal recognition protocol (SRP) antibody	Negative
Jo-1 (histidyl-tRNA synthetase)	1 AU/mL
Ku antibody	Negative
Smith/RNP (ENA) IgG antibody	9 unit(s)
SSA-52 (Ro52) (ENA) IgG antibody	Negative
SSA-60 (Ro60) (ENA) IgG antibody	1 AU/mL
Fibrillarin (U3 RNP) IgG antibody	Negative
PM/Scl-100 antibody	Negative

The patient was diagnosed by our consultant rheumatologist with necrotizing immune-mediated myositis caused by statin therapy. She was treated with intravenous immunoglobulin and steroids with significant improvement. A muscle biopsy was obtained and the pathologist reported the following: an examination of sections revealed skeletal muscles with severe necrotizing myopathy, mild chronic inflammation, MHC class-I staining necrotic fibers, and rare staining of non-necrotic fibers. The mildly increased fibrosis suggested the findings may be at least subacute to chronic. The markedly elevated CPK was concordant with severe necrotizing myopathy. Multiple entities were on the differential with statin-induced myopathy (frequently secondary to anti-hydroxymethylglutaryl-coenzyme A reductase antibody with immune-mediated necrotizing myopathy) as a distinct possibility. Findings were somewhat more severe than often seen with statin-induced myopathy but they can be this severe. Steroid therapy can mask inflammatory myopathies and additional underlying inflammatory myopathy was not excluded. There was moderate fiber type II atrophy possibly due to disuse and or steroid therapy or other etiology. Significant neurogenic findings were not identified. The pathologist reported that this represents severe necrotizing myopathy with steroid therapy possibly masking other inflammatory myopathies. The findings were compatible with statin-induced myopathy even if they were somewhat in the severe range for this entity. Written consent from the patient was obtained to publish this case report.

The article "Statin-Induced Autoimmune Necrotizing Myositis: A Case Report" was published in 2022. Journal: Cureus.

## Discussion

This patient was prescribed high-dose rosuvastatin 40 mg once daily as part of her guideline-directed medical therapy for her coronary artery disease with percutaneous intervention. The patient was taking her medication for about four months before admission. The patient reported some muscle pain when the medication was started. However, it worsened in the period prior to admission. Worsening of myopathy or the development of an autoimmune response to statin therapy can occur after long-term use.

We suspected that the patient had statin-related muscle weakness as her CPK was significantly elevated on admission. MRI of the thighs showed symmetric edema within the musculature of the proximal to mid-thighs which is due to inflammatory response and necrosis. Dermatomyositis and polymyositis were excluded because the patient did not have a rash or upper extremity weakness. Other differentials include anti-signal recognition peptide antibody; however, this is usually accompanied by dysphagia which the patient did not have. Other myositis-inducing antibodies were negative and were less likely to be the cause of her myositis. The patient reported improvement in symptoms after the statin was stopped, and she received intravenous immunoglobulin [3,4]. This improvement in symptoms after stopping the offending agent also points to the likelihood that her necrotizing myositis was statin-induced though we agree that most of her rapid improvement was due to steroid therapy. The patient has done well since the discontinuation of her statin in multiple follow-ups with no repeated episodes of myositis ruling out other autoimmune disease processes that would have otherwise recurred regardless of statin therapy.

## Conclusions

Statin-induced autoimmune necrotizing myositis can be a side effect that presents at a later time during therapy due to antibodies forming against the hydroxymethylglutaryl-coenzyme A reductase which mainly affects the muscles. Statin therapy remains one of the cornerstones of therapy in coronary artery disease patients. Discontinuation of therapy might not be enough to resolve symptoms, and patients might need immunosuppressive therapy.
